The article "Intelligent Algorithm-Based Electrocardiography to Predict Atrial Fibrillation after Coronary Artery Bypass Grafting in the Elderly" was published in 2022. Journal: Comput Math Methods Med.

# Intelligent Algorithm-Based Electrocardiography to Predict Atrial Fibrillation after Coronary Artery Bypass Grafting in the Elderly

**DOI:** 10.1155/2022/4596552

**Published:** 2022-03-09

**Authors:** Tao Feng, Zhihua Deng

**Affiliations:** Department of Cardiovascular Medicine, Zhongshan People's Hospital, Zhongshan 528400, China

## Abstract

The objective of this study was to explore the predictive value of electrocardiogram (ECG) based on intelligent analysis algorithm for atrial fibrillation (AF) in elderly patients undergoing coronary artery bypass grafting (CABG). Specifically, 106 elderly patients with coronary heart disease who underwent CABG in the hospital were selected, including 52 patients with postoperative AF (AF group) and 54 patients without arrhythmia (control group). Within 1-3 weeks after operation, the dynamic ECG monitoring system based on Gentle AdaBoost algorithm constructed in this study was adopted. After the measurement of the 12-lead P wave duration, the maximum P wave duration (Pmax) and minimum P wave duration (Pmin) were recorded. As for simulation experiments, the same data was used as the back-propagation algorithm. The results showed that for the detection accuracy of the test samples, the Gentle AdaBoost algorithm showed 93.7% accuracy after the first iteration, and the Gentle AdaBoost algorithm was 16.1% higher than the back-propagation algorithm. Compared with the control group, the detection rate of arrhythmia in patients after CABG was significantly lower (*P* < 0.05). Bivariate logistic regression analysis on Pmax and Pmin showed as follows: Pmax: 95% confidential interval (CI): 1.024-1.081, *P* < 0.05; Pmin: 95% CI: 1.036-1.117, *P* < 0.05. The sensitivity of Pmax and Pmin in predicting paroxysmal AF was 78.2% and 73.4%, respectively; the specificity of them was 80.1% and 85.6%, respectively; the positive predictive value was 81.2% and 83.4%, respectively; and the negative predictive value was 79.5% and 75.3%, respectively. In conclusion, the generalization ability of Gentle AdaBoost algorithm was better than that of back-propagation algorithm, and it can identify arrhythmia better. Pmax and Pmin were important indicators of AF after CABG.

## 1. Introduction

Atrial fibrillation (AF) is a common kind of arrhythmia. Arrhythmia refers to the abnormal speed and uniformity of heart beating and mainly manifests as too fast, too slow, or irregular heart beating [1, 2]. When AF occurs, the rapid and irregular electrical signals will cause the fibrillation of the right ventricle and the left atrium so that they cannot contract normally, the blood in the atrium cannot all enter the ventricle, and the atrium and ventricle cannot coordinate normally [3]. AF affects 2.5 million people in the United States, 4.5 million in the European Union, and more than 8 million in China. The cumulative incidence was 2.2% in males and 1.7% in females. AF shows a higher incidence in patients with heart failure and valvular disease, and about 70% of AF is secondary to patients with organic heart disease. In addition, it is easy to occur during the perioperative period of coronary artery bypass grafting (CABG) [4–6]. At present, the pathogenesis of AF is not clear. The main reason is the abnormal atrial muscle structure caused by heart or systemic diseases, leading to atrial remodeling or atrial muscle ischemia. Medical studies have confirmed that AF is related to age, CABG, heart disease, blood transfusion, and chronic diseases [7].

The article "Intelligent Algorithm-Based Electrocardiography to Predict Atrial Fibrillation after Coronary Artery Bypass Grafting in the Elderly" was published in 2022. Journal: Comput Math Methods Med.

The diagnosis of AF mainly includes the electrocardiography (ECG) examination and physical examination. ECG refers to the heart wave curve recorded by placing the guiding electrode on the surface of the body [8–10]. In every cardiac cycle, the excitatory signal from antrum room node is spread in a fixed way to atrium and ventricle so that the whole heart is excitatory. The excitation can induce bioelectric changes in the conduction process which then spread to the whole body through the conductive cell and humoral fluid. Accordingly, in every cardiac cycle, all parts of the body surface will produce regular electrical signals [11]. Parsi's [12] team described a method based on finding and counting multiple types of repetitive features in atrial fibrillation cycle waveform, and applying means to classify them, so as to achieve high accuracy prediction of atrial fibrillation. P wave is the atrial depolarization wave generated in the depolarization process of left atrium, right atrium, and atrial septum, which can fully reflect the potential changes of the excitation signal in the atrial conduction process. The generation of ECG depends on the bioelectrical changes of cardiomyocytes, and the cardiomyocyte electrical activity on the body surface becomes the potential value at each moment of electrocardiogram, and the two are closely related [13].

ECG is a recognized method in the medical field to diagnose AF. However, most ECG physicians in China today are inexperienced, and there are very few doctors who can read ECG skillfully and accurately [14]. Additionally, the reliability of automatic diagnosis of most 12-lead ECGs is still very low [15, 16]. Therefore, a more effective method is urgently needed to complete the automatic recognition of ECG. With the rapid development of the computer intelligence technology, the Gentle AdaBoost algorithm has made great achievements in the medical field and has been widely used in the diagnosis and treatment of cardiovascular and cerebrovascular diseases [17].

The article "Intelligent Algorithm-Based Electrocardiography to Predict Atrial Fibrillation after Coronary Artery Bypass Grafting in the Elderly" was published in 2022. Journal: Comput Math Methods Med.

The innovation of this work was the Gentle AdaBoost algorithm-based ECG. First, the characteristics of the ECG were extracted, and then, the classification model was trained by deep learning. Finally, the trained model was used to automatically identify the premature ventricular contract (PVC) of AF after CABG in 106 elderly patients, aiming to analyze the predictive value of ECG based on Gentle AdaBoost algorithm for AF after CABG in elderly patients.

## 2. Materials and Methods

### 2.1. Research Subjects

In this study, 106 elderly patients with coronary heart disease in the hospital from November 20, 2018, to May 20, 2020, were selected, including 58 males and 48 females, with an average age of 62.35 ± 9.64 years old. Of the 106 elderly patients, there were 52 patients with new atrial fibrillation after CABG (AF group) and 54 patients without CABG (control group). This study had been approved by the committee of hospital, and patients and their families had understood the research situation and signed the informed consent form.

Inclusion criteria are as follows: (1) patients with no AF before CABG, (2) patients with no postoperative hypokalemia, (3) patients aged over 55, and (4) patients whose AF was detected by the dynamic body surface ECG.

Exclusion criteria are as follows: (1) patients whose AF was caused by electro-physiological examination and cardiac angiography, (2) those accompanied by severe infections and trauma, (3) those complicated with malignant tumors, (4) those with incomplete ECG data, and (5) those combined with cardiomyopathy, aortic dissection, and congenital heart disease.

### 2.2. The ECG Data Acquisition Method

All the patients with coronary heart disease were monitored dynamically for 24 hours by ECG monitoring system based on Gentle AdaBoost algorithm within 1-3 weeks after CABG. The paper speed was 25 mm/s, and the gain was 10 mm/Mv. Then, they were manually detected. The computer analysis results of reference instruments and referring to the patient's life records were adopted to form a result report.

### 2.3. Data Measurement and Its Standard

The ECG measuring software was used to measure the P wave duration of each lead in the ECG of the 52 elderly patients with coronary heart disease.  Figure 1 shows the width (s) and amplitude (mm) of the negative part of the P wave terminal potential of lead V1 (PTFV1). The measurement standards are as follows. The starting point of P wave measurement is at the intersection of P wave starting point and equipotential line, and the end point of P wave measurement is at the intersection of P wave ending point and equipotential line. The time limit of P wave in each lead is measured separately with a stable heart cycle at baseline, and three P waves with clear graphics are continuously measured in each lead, and the average value is taken as the time limit of P wave in that lead. After the 12-lead P wave time limit was measured, the longest and shortest time limit refers to the maximum P wave duration (Pmax) and the minimum P wave duration (Pmin), respectively.

The article "Intelligent Algorithm-Based Electrocardiography to Predict Atrial Fibrillation after Coronary Artery Bypass Grafting in the Elderly" was published in 2022. Journal: Comput Math Methods Med.

### 2.4. ECG Based on Gentle AdaBoost Algorithm

The intelligent analysis of ECG mainly includes three steps: pretreatment of ECG, feature extraction of ECG, and ECG analysis.  Figure 2 shows the flowchart of ECG based on Gentle AdaBoost algorithm. ECG pretreatment mainly included ECG filtering, removing 55 Hz power frequency interference, and correcting baseline drift. Feature extraction required to locate the P wave peak first and then calculate the wave group width and other characteristic parameters step by step. The ECG analysis in this work focused on automatic recognition of PVC. PVC refers to the arrhythmia ventricular premature beat. It occurs when the sinus excitation has not been transmitted to the ventricle; a pacemaker in the ventricle is excited in advance, leading to ventricular depolarization. Long-term ECG monitoring of PVC can predict cardiac abnormalities and prevent them from happening.

In this work, Gentle AdaBoost algorithm is used to construct a strong classifier to classify ECG. One is arrhythmia, and the other is other categories. In this work, R peak is extracted by wavelet transform, and six positions of P wave, Q wave, Q wave, S wave, S wave, and T wave are extracted. The Gentle AdaBoost algorithm was described as follows [18].

For the given *m* abnormal training samples, (X1,Y1)..., (Xm,Ym), Yi ∈ {−1, +1}, and -1 represents PVC, and +1 represents other arrhythmia types. The weight of the initialization training sample was Wi = 1/*m*, (1, 2, 3, ⋯, *m*), and the classifier met *F*(*X*) = 0. For all the input samples, the most suitable weak classifier *FN* (*X*) was found after *n* times, so that the mean error of samples was the minimum, and then, *F*(*X*) + *fn*(*X*)⟶*F*(*X*) was updated. Next, the weight Wiexp(−Yifn(Xi))⟶Wi of the sample was updated and unified to meet ∑_*i*=1_^*m*^Wi = 1.Finally, a strong classifier *F*(*X*) = sign(∑_*n*=1_^*N*^*fn*(*X*)) was obtained.

### 2.5. Simulation Experiment of the Gentle AdaBoost Algorithm-Based ECG

1242 arrhythmias were collected from the MIT-BIH ECG database in this work, of which 254 were PVCs, 854 were normal beats, and the rest were other types of arrhythmias. The same data was used for simulation experiments in this work to verify the performance of the Gentle AdaBoost algorithm. In this study, MATLAB is used to simulate the BP algorithm of neural network and Gentle AdaBoost algorithm, with 621 data as training samples and another 621 data as test samples. There were 124 cases of PVC in the training samples and also 105 cases of PVC in the test samples. Then, the simulation experiment was conducted after the exchange of training samples and test samples. The input node of the back-propagation algorithm was 10, the output node was 2, the learning rate was set as 0.2, and the variance of the target mean was 0.002. The number of iterations of the Gentle AdaBoost algorithm was set to 100.

The article "Intelligent Algorithm-Based Electrocardiography to Predict Atrial Fibrillation after Coronary Artery Bypass Grafting in the Elderly" was published in 2022. Journal: Comput Math Methods Med.

The hardware configuration and software configuration of the test environment in this work were defined as follows. The server is Windows Server 2013 server, the processor is i7, the memory is 2G, the main frequency is 2.6 GHz, a 100 M network card is added, and the access bandwidth is 2 M. The operating system is Windows Server 2013, and the database version is SQL Server 2015. The server side is a web site, and a Windows IIS server is used to set up the web site.

### 2.6. Evaluation Methods

Two experienced ECG clinicians in hospital diagnosed the cardiac rhythm status of patients with coronary heart disease according to ECG results. If the two physicians have the same diagnosis, that is the gold standard. In case of inconsistency, a third expert could be invited for arbitration. Next, the unified results of the three experts were taken as the gold standard. Then, the results of the Gentle AdaBoost algorithm were compared with the gold standard to evaluate the accuracy of the Gentle AdaBoost algorithm in detecting arrhythmia.

### 2.7. Statistical Methods

SPSS 21.0 was used for statistical analysis of the data. The calculated data conforming to normal distribution were represented by the mean ± standard deviation (−*X* ± *S*), and the *t*-test was adopted. The nonconforming data were expressed as the percentage (%), and *χ*^2^ test was used. Binary logistic regression was used for multivariate analysis, and receiver operating characteristic (ROC) curve was used to evaluate the predictive value of related indicators for AF after CABG. *P* < 0.05 indicated significant differences.

## 3. Results

### 3.1. Simulation Results of Back-Propagation and Gentle AdaBoost Algorithms

In the simulation experiment, the error of the back-propagation algorithm and the Gentle AdaBoost algorithm on the training samples was both 0. For the detection accuracy of test samples, the back-propagation algorithm got 82.1% accuracy after the first iteration. The Gentle AdaBoost algorithm got 93.7% accuracy after the first iteration and got two weak classifiers. The accuracy rate of Gentle AdaBoost algorithm is 11.6% higher than that of back propagation algorithm, as shown in Figure 3. The simulation results suggested that the generalization ability of the Gentle AdaBoost algorithm was better than that of the back-propagation algorithm. Faced with the ever-changing ECG waveform, the Gentle AdaBoost algorithm can better identify arrhythmia.

The article "Intelligent Algorithm-Based Electrocardiography to Predict Atrial Fibrillation after Coronary Artery Bypass Grafting in the Elderly" was published in 2022. Journal: Comput Math Methods Med.

### 3.2. Baseline Data of Patients in Both Groups

In the AF group, there were 52 patients, with an average age of 63.87 ± 8.85 years and an average weight of 76.28 ± 8.27 kg. Of the 52 patients, there were 25 male patients (48.1%), 27 female patients (51.9%), 24 smoking patients (46.2%), 25 drinking patients (48.1%), 24 diabetes patients (46.2%), 27 cases (51.9%) with hypertension, 25 cases (48.1%) with myocardial infarction, and 41 cases (78.9%) with three-vessel disease. In the control group, there were 54 patients, with an average age of 61.25 ± 7.12 years and an average body weight of 78.15 ± 9.21 kg. Of the 54 cases, there were 33 male patients (61.1%), 21 female patients (38.9%), 25 smoking patients (46.3%), 26 drinking patients (48.1%), 26 diabetes patients (48.2%), 28 cases (51.9%) with hypertension, 25 cases (46.3%) with myocardial infarction, and 43 cases (79.6%) with three-vessel disease. There was no statistical difference in preoperative basic data of patients between the two groups (*P* > 0.05), as shown in Table 1 and Figure 4.

### 3.3. Detection Rate of Arrhythmia

Of the 52 patients with cardiac arrhythmia after CABG, the incidence of supraventricular arrhythmia was the highest (86.5%), followed by AF (19.2%). Both the supraventricular speed and ventricular tachycardia were short paroxysmal, as shown in Figure 5. There were 3 patients who could not recover the autonomic rhythm during the operation and required temporary pacemaker, 5 having pacing for 2 days, 2 having pacing for 3 days, and 1 with recovered autonomous cardiac rhythm after 3 weeks. Compared with the control group, the detection rate of arrhythmia after CABG was significantly reduced (*P* < 0.05).

### 3.4. Multivariate Analysis of AF and Control Groups

The univariate analysis results of statistically significant indicators (gender, Pmax, Pmin, P wave terminal potential of lead V1 (PTFV1), and anterior-posterior diameter (LAD)) were analyzed by binary logistic regression. The results showed that Pmax, Pmin, and PTFV1 were important indicators to predict the occurrence of postoperative AF (Pmax: 95% CI: 1.024-1.081, *P* < 0.05; Pmin: 95% CI: 1.036-1.117, *P* < 0.05; PTFV1: 95% CI: 0.000-0.402, *P* < 0.05) (Table 2).

The article "Intelligent Algorithm-Based Electrocardiography to Predict Atrial Fibrillation after Coronary Artery Bypass Grafting in the Elderly" was published in 2022. Journal: Comput Math Methods Med.

### 3.5. Predictive Value of Pmax, Pmin, and PTFV1 for AF after CABG

ROC curve was used to evaluate the predictive value of Pmax and Pmin for paroxysmal AF. The results showed that the area under the curve of Pmax was 0.892 to predict the occurrence of postoperative AF. The optimal critical value was determined by Youden index to be 125.7 ms, and Pmax ≥ 125.7 ms. The sensitivity, specificity, positive predictive value, and negative predictive value of Pmax to predict the occurrence of paroxysmal AF were 78.2%, 80.1%, 81.2%, and 79.5%, respectively. The area under the curve (AUC) of Pmin was 0.823 to predict the occurrence of postoperative AF, and the optimal critical value was determined by Youden index to be 108.5 ms, and Pmin ≥ 108.5 ms. The sensitivity, specificity, positive predictive value, and negative predictive value of Pmin to predict the occurrence of postoperative AF were 73.4%, 85.6%, 83.4%, and 75.3%, respectively. The AUC of PTFV1 for predicting paroxysmal atrial fibrillation was 0.628, and the best critical value determined by Joden index was -0.015 mm s. The sensitivity, specificity, positive predictive value, and negative predictive value of PTFV1 ≤ −0.015 mm s for predicting paroxysmal AF were 61.3%, 72.8%, 67.2%, and 63.6%, respectively (Table 3 and Figure 6).

## 4. Discussion

AF is a common kind of arrhythmia, and its incidence is increasing in recent years. There are many influencing factors of AF after CABG, including systemic hypokalemia, hyperthyroidism, cardiac valvular disease, heart failure, and ischemic heart disease [19, 20]. The incidence of AF after CABG is high, and it can be quickly diagnosed according to clinical manifestations, signs, and ECG [21]. For a long time, ECG has been the most commonly used method for diagnosing and screening AF in clinic [22]. Traditional ECG data mostly rely on manual feature extraction, and the subjectivity is high. For example, the results are not accurate when they feel fatigue due to long time work, reducing the reliability of ECG report. Moreover, arrhythmias in many patients have no obvious rules, often one-time or intermittent, and some only appear at night without obvious clinical manifestations, which cannot be accurately captured by traditional ECG. With the continuous development of computer intelligence technology, ECG automatic analysis system is gradually applied in China. In this work, the patients were monitored by Gentle AdaBoost algorithm-based ECG continuously to accurately identify all kinds of arrhythmias, assisting clinicians in effective and accurate reading of ECG [23].The diagnosis results of ECG by 2 electro-cardiologists were used as the gold standard to evaluate the accuracy of Gentle AdaBoost algorithm in monitoring arrhythmias. The results showed that the incidence of supraventricular arrhythmia was the highest (86.5%), followed by AF (19.2%), and both supraventricular tachycardia and ventricular tachycardia were short parturient. Such results suggest that the Gentle AdaBoost algorithm-based ECG can meet the requirements for detecting supraventricular arrhythmia and AF, which is consistent with the research results of Yanagisawa et al. [24].

The article "Intelligent Algorithm-Based Electrocardiography to Predict Atrial Fibrillation after Coronary Artery Bypass Grafting in the Elderly" was published in 2022. Journal: Comput Math Methods Med.

Compared with the control group, the detection rate of arrhythmia after CABG was significantly reduced (*P* < 0.05). This suggests that after CABG, blood supply to myocardium is significantly improved, and some or all functions of myocardial cells are restored. After revascularization of the right coronary artery, the incidence of supraventricular arrhythmia was significantly reduced.

Pmax and Pmin are important indicators to predict the occurrence of postoperative AF (Pmax: 95% CI: 1.024-1.081, *P* < 0.05; Pmin: 95% CI: 1.036-1.117, *P* < 0.05). The internal mechanism of the prediction of Pmax and Pmin on postoperative AF is mainly that P wave duration represents the time of atrial depolarization. When the electrical signals in the left and right heart rooms and single atrial are abnormal, it will lead to atrial electrical remodeling, which is manifested as prolonged P wave duration in electrocardiogram. AF itself can lead to atrial enlargement, atrial structural remodeling, and systolic remodeling. When atrial enlargement is abnormal, cardiac ECG vector will change significantly, which is the main factor leading to the increase of absolute values of Pmax and Pmin. The AUC for Pmax to predict the occurrence of postoperative AF was 0.892. The optimal critical value was determined by Youden index to be 125.7 ms, and Pmax ≥ 125.7 ms. The AUC for Pmin to predict the occurrence of postoperative AF was 0.823, and the optimal critical value was 108.5 ms using Youden index. The optimal critical value in this work was superior to the traditional critical value obtained by Eerikäinen et al. [25] in terms of the predictive ability of AF.

## 5. Conclusion

With the improvement of people's living standard and education level, people gradually realize the importance of health, and the demand for medical conditions and services increases accordingly. In this work, ECG based on the Gentle AdaBoost algorithm was constructed to predict the occurrence of AF in 106 elderly patients with coronary heart disease undergoing CABG. The generalization ability of the Gentle AdaBoost algorithm was found to be better than that of the back-propagation algorithm. In the face of the changing ECG waveform, the Gentle AdaBoost algorithm can better identify arrhythmia. Pmax and Pmin were proved to be important indicators of AF after CABG. The shortcoming of this work was that the quality of the included ECG data was different, which increased the measurement error in P wave duration and amplitude. In addition, it was a single-center study with a small sample size, so it was necessary to expand the sample size and include high-quality data for in-depth discussion in the later stage. All in all, ECG is simple to operate and low in cost. Choosing the best prediction index can provide clinicians with early warning of atrial fibrillation after coronary artery bypass grafting. I hope that it can better serve the clinic in the future and help clinicians to complete clinical practice more efficiently.

The article "Intelligent Algorithm-Based Electrocardiography to Predict Atrial Fibrillation after Coronary Artery Bypass Grafting in the Elderly" was published in 2022. Journal: Comput Math Methods Med.

## Figures and Tables

**Figure 1:** Schematic diagram of P wave duration. P represents the exciting process of left and right atria; QRS is the part of electrocardiographic wave, which reflects the potential changes of two ventricles during the propagation of excitement; PR is the time interval from the wave starting point to the wave group starting point; T is a waveform with a longer band and lower amplitude after QRS complex; ST refers to the waveform from the end of S wave to the beginning of T wave; QT refers to the waveform from the end of Q wave to the beginning of T wave.

**Figure 2:** ECG based on Gentle AdaBoost algorithm.

**Figure 3:** Accuracy rate of the back-propagation and Gentle AdaBoost algorithm. ^∗^ represented significant difference compared with back-propagation algorithm (*P* < 0.05).

**Figure 4:** Comparison of baseline data between the two groups: (a) sex, smoking, and drinking; (b) diabetes mellitus, hypertension, myocardial infarction, and three-vessel disease.

**Figure 5:** Comparison of arrhythmias between the two groups: (a) comparison of sinus rhythm, sinus bradylosis, sinus tachycardia, sinus arrest, and AF; (b) comparison of ventricular tachycardia, supraventricular speed, and PVC. ^∗^ represented significant difference compared with the AF group (*P* < 0.05).

**Figure 6:** ROC curves of Pmax and Pmin to predict postoperative AF.

**Table 1:** Comparison of age and weight between atrial fibrillation group and control group.

Project	AF group	Control group	*t* value	*P* value
Age (years)	63.87 ± 8.85	61.25 ± 7.12	1.895	0.062
Weight (kg)	76.28 ± 8.27	78.15 ± 9.21	12.438	0.053

**Table 2:** Multivariate logistic regression analysis of patients with and without AF.

Variable	Mean deviation	Wald value	*B* value	OR value	95% CI	*P* value
Pmax (ms)	0.015	22.324	0.067	1.047	1.024-1.081	<0.05
Pmin (ms)	0.017	28.417	0.084	1.084	1.036-1.117	<0.05
PTFV1 (mm·s)	6.317	5.261	-13.21	0.000	0.000-0.402	<0.05

The article "Intelligent Algorithm-Based Electrocardiography to Predict Atrial Fibrillation after Coronary Artery Bypass Grafting in the Elderly" was published in 2022. Journal: Comput Math Methods Med.

**Table 3:** The predictive value of Pmax and Pmin for the occurrence of postoperative AF.

Variable	AUC	95% CI	Sensitivity (%)	Specificity (%)	Positive predictive value (%)	Negative predictive value (%)	The optimal critical value (%)
Pmax (ms)	0.892	0.852-0.912	78.2	80.1	81.2	79.5	125.7
Pmin (ms)	0.823	0.715-0.834	73.4	85.6	83.4	75.3	108.5
PTFV1 (mm·s)	0.628	0.587-0.653	61.3	72.8	67.2	63.6	-0.015

## Data Availability

The data used to support the findings of this study are available from the corresponding author upon request.
